# Urban Landscaping Landscape Design and Maintenance Management Method Based on Multisource Big Data Fusion

**DOI:** 10.1155/2022/1353668

**Published:** 2022-08-30

**Authors:** Lijuan Zhu

**Affiliations:** Zhengzhou University of Aeronautics, Henan, Zhengzhou 450046, China

## Abstract

In the process of continuous urbanization construction, the construction scale of urban landscaping projects is getting larger. At the same time, the design and the maintenance of the management is becoming more important. Recently, the rocketing development of the ternary world of many people, machines, and things has triggered the generation of multisource fusion data and the development of artificial intelligence technology, and the world has entered the era of multisource big data intelligence. Multisource data refer to the fusion of multiple types of data with effective characteristic information, which has richer, more comprehensive, more detailed, and more effective information than a single data source, and can provide high-quality data sources for various complex problems. Therefore, more effective data can be provided for the definition of urban fringe areas. From the moment Google's AlphaGo defeated Go world champion Li Shishi, the chess game has been occupied by AI, setting off an upsurge in the study, research, and application of AI technology. Colleges and universities around the world have followed suit and set up AI-related majors. Deep learning is one of the cutting-edge technologies in the field of artificial intelligence. It is a method to solve complex real-life problems by extracting effective information from the data and mining key features on the basis of a large amount of learning and computing data.

## 1. Introduction

Landscaping landscape design is a thinking process and planning strategy for people with relevant professional knowledge of architecture, plants, aesthetics, literature, etc. to consciously transform the natural environment on the basis of traditional garden theory. Specifically speaking, this is the procedure of building a beautiful and natural environment as well as the living and recreational environment within the scope of geography, employing the garden art and engineering techniques, or over transforming terrain, planting plants, creating buildings, and arranging garden roads. Through landscape design, the environment has aesthetic appreciation value, daily use function, and can ensure ecologically sustainable development [1].

The construction of urban garden landscapes in various places has become a very important content in urban construction. Whether urban landscape planning can adapt to the development and requirements of urban construction, and how to meet the needs of urban residents, will become an important measure of “livability” [2]. As a kind of human landscape, the urban garden landscape is a complex natural landscape and artificial landscape. To achieve the ideal realm of “living in a poetic place,” the ideal realm of “original” urban landscape must be carried out, and an “original” urban landscape design must be carried out to maximize the value of the landscape [3]. Under the background of advocating a conservation-oriented society and a harmonious society, both urban landscape and small and medium-sized town landscape construction should take regionality as the most basic principle and explore the design methods of preserving culture, continuing history, and saving resources.

In landscape design, we should obtain a larger green area and a better landscape design effect with less investment [4]. Therefore, the original ecological elements should be fully respected in the design, and the original terrain, vegetation, and other elements should be used as much as possible to achieve the design purpose. Interpret the site from the regional scale, analyze the landscape characteristics of the existing urban built-up area and the relationship between the site and the surrounding environment, and grasp the context and direction of development. The comprehensive site analysis includes the analysis of the natural elements, regional characteristics, and cultural landscape of the site. The comprehensive analysis of the site is actually a process of finding and interpreting the landscape and reading the Earth. On the basis of a full investigation of various elements, a comprehensive analysis is carried out, and favorable factors, unfavorable factors, and development potentials are proposed. A detailed site analysis can effectively provide guidance for planning. For example, in reality, in expressing the mountain and rock scenery, the original stones and plants on the site can be used and modified in the later stage to make the original scenery more in line with the design idea.

Urban landscape protection design must follow the protection of natural landscape, and strictly speaking, it is ecological design. Eco-city natural relics contain representative samples of biological communities and landscapes, and the animal and plant species, habitats, and landforms in them are of significance for conservation, education, recreation, and popular science. According to different management purposes, it can be further divided into ecological protection type, ecological tourism type, ecological science popularization type, and so on. In urban landscape design and construction, biodiversity is a factor that must be considered. The urban landscape is an indispensable part of people's life and production. In urban landscape design, the positive and negative impacts of landscape design on biodiversity and the ecological environment must be considered. The protection design of the architectural landscape must fully consider the optimal use of resources. In the overall design of the city, the rational use of resources is the most important. Replacing all the old to meet the new requirements is wasteful and expensive, destroying entire cities or even a region. We must break the balance somewhere, take the scientific concept of development as the guide, combine the local reality, and at the same time refer to the experience of other places, and do a good job in the protection of the urban landscape.

The multisource data fusion method is originated in the 1960s. It refers to the technology of using relevant means to integrate all the information obtained from investigation and analysis, evaluate the information uniformly, and finally obtain unified information. The purpose of this technology is to synthesize various different data information, absorb the characteristics of different data sources, and then extract unified, better, and richer information than single data. Compared with the single data source model, the multisource data model has more original information and is better in data inference. Dana argues that, in many disciplines, information can be obtained from a variety of sources, including different types of measurement instruments, different measurement techniques, and different experimental setups. Due to the complexity of some natural courses, it is not possible for a single exploring method to present an all-rounded comprehension of them. In natural life, we humans perceive things through various senses. We have hearing, sight, smell, taste, etc. to perceive everything in the world. Various senses in our body acquire information about a phenomenon, and then, each sense transmits the acquired information to the brain, and finally, the brain integrates the information transmitted by various sensory parts to make judgments about things. Covers specific information in the area, and finally, transmits this information to the owner of the network. At present, the number of samples involved in most data fusion literature is relatively small. In large sensor networks, due to a large number of sensor nodes, if each sensor node carries a large amount of data, processing data from all sensors is a big task, facing a huge amount of computation.

## 2. Materials and Methods

Foreign scholars have a wide range of research fields on the fusion of multisource datasets. After collecting data from different nodes, we must consider whether the data are affected specifically by each node before modeling the data. Since data sets from different sources may have problems such as distribution shifts and inconsistent measurement standards, it is not possible to directly integrate all data together. Due to the problems of distribution shift and nonuniform measurement standards in the datasets from different sources, it is not possible to directly integrate all the data together. At present, most statistical machine learning research has proposed some algorithms to solve the distribution shift or perform data fusion [6, 7]. For example, Ben-David and Schuller pointed out that domain adaptation problems involving data set or covariate transfer should first align the data distribution for further data analysis [8]. Such algorithms usually suffer from bias in the sampling process, which is generally solved by weighting [9]. The literature on domain adaptation focuses on using a certain type of algorithm to solve the problem of differences between nodes before fusing the data, and after eliminating the differences between different data sets, is it significant to fuse the data together? Zhou et al. considered the integration of data sets from two different places, established a linear regression model in the case of small samples, and proposed hypothesis testing in the case of small samples. And combined with real datasets, it is demonstrated that fusing together similar datasets from multiple sites improves the statistical power of the model [10]. Zhou et al. used a graphical model approach to address the problem of distribution transfer in different datasets and proposed a hypothesis test under which conditions such datasets can be fused or analyzed. And using the support vector machine method, combined with the Alzheimer's disease dataset, the classification problem of the fused dataset is considered. Due to the particularity of some diseases, the number of patients is relatively small, and the amount of related data is also small [11]. Dana Lahat et al. proposed a multimodal data fusion method to fuse datasets obtained by different means [12]. D. L. Hall compares multisensor data fusion with single sensor data fusion and believes that multisensor data fusion will have more advantages in data accuracy and practical application. In addition, in terms of information presentation and expression, multisource and multimodal data also increase robustness. For example, audio does not need a line of sight, and video is not afraid of environmental noise. Therefore, when there are high requirements for information quality, such as the high requirements for accuracy of medical diagnosis and the comprehensive requirements of meteorological prediction for data, the fusion and integration of multisource data are an important basis for improving the quality of data analysis. Domestic research on multisource data fusion started relatively late, but it has developed rapidly in the past two years. Fang Kuangnan and Zhao Mengmi selected data from two sources, rural and urban, and proposed a logistic regression model based on multisource data fusion for personal credit scoring. The results of the study show that the prediction effect of the integrated model is better than that of the independent dataset model [13]. Xiong Lifang and Zhen Feng used Baidu index to obtain user attention data among cities in the Yangtze River Delta and analyzed the temporal and spatial evolution characteristics of cities in the Yangtze River Delta by simulating urban information flow [14]. Shi Lina used the five-year road passenger and freight volume data of 133 counties in two provinces and one city in the Yangtze River Delta for analysis and judged the changes and grades of node cities through the spatial connection reflected by road passenger and freight volumes [15].

Compared with the traditional way of obtaining data through research, the technology of big data is featured by the large volume, timely and microscopic information. With the emergence of big data sources such as social media, online media, and mobile communications, the application of big data has broken through the space, and the shackles of the time category, the laws of human behavior, and the social attributes of the garden environment have been paid more attention by researchers [16]. The research objects cover the landscape architecture environment of various types and scales, such as urban green space, ecological service facilities, and scenic spots [17]. Through computer software and algorithms and other technologies to analyze mobile phone positioning data, map service POI data, social network data, traffic sensor data, and other open data, to solve space quality assessment, greenway planning, location and route selection, and green space usage rules and related issues such as the assessment of influencing factors. With the breaking down of big data acquisition barriers and the maturity of data mining and processing technologies, the precision and accuracy of big data analysis will be significantly improved [18].

## 3. Results and Discussion

### 3.1. 3D Urban Garden Landscape Generation

Texture path selection is quite important in improving the vraisemblance of the texture. In the process of the 3D garden landscape, the problems are disguised as the best path in the condition of multiconvergence [19].

The paper will get rooted in the practical problems and explicit the spatial scale. The weighing adjacency which can express the best problem range will be given. In this process, the characteristic points on each path of the whole graph were marked with the optimal problem scale for simulated ants, and the individual ants were marked [20–23].

The pheromone should be updated after the ants traverse a complete cycle to avoid the problem, which can be changed by the following formula:

(1) $$\begin{array}{c} \tau_{ij}\left(t+n\right)=\left(1-\rho \right)\cdot \tau_{ij}\left(t\right)+\Delta \tau_{ij}\left(t\right), \end{array}$$

(2) $$\begin{array}{c} \Delta \tau_{ij}\left(t\right)=\sum_{k=1}^{m}\Delta \tau_{ij}^{k}\left(t\right). \end{array}$$

The fixed information pheromone volatility element is indicated by *p*, and the total number of the setting ant colonies which is optimized by the scale of the problems is shown as *m*. Basically, if the value of *m* is even higher, the possibility of the best results will be better acquired. The update process is

(3) $$\begin{array}{c} \Delta \tau_{ij}^{k}=\left\{\begin{array}{cc} Q/C^{K}, & \text{Path}\left(i,j\right)\text{Be traversed by ants,}\\ 0, & \text{Other circumstances.} \end{array}\right. \end{array}$$

### 3.2. Information Fusion Model Construction

GA takes the fitness function as the evolutionary target which is assumed that the population size is *N*, the individual in the population is FI, *F* (*F*_*i*_) represents the individual fitness value, and the selection probability *P*_*i*_ is calculated as follows:

(4) $$\begin{array}{c} P_{i}=\frac{F\left(f_{i}\right)}{\sum_{i=1}^{N}F\left(f_{i}\right)}. \end{array}$$

First calculate the cumulative probability Pi:

(5) $$\begin{array}{c} P_{i}=\sum_{i=1}^{N}p_{i},\;i=1,2,\ldots ,N. \end{array}$$

In order to prevent premature convergence, the adaptive *P*_*c*_ and *P*_*d*_ methods are used. *P*_*c*_ and *P*_*d*_ are changed according to the adaptive function of the solution. The process is as follows:

(6) $$\begin{array}{c} P_{c}=\left\{\begin{array}{cc} \left(f_{\max}-f^{\prime }\right)\left(f_{\max}-f_{\text{avg}}\right), & f^{\prime }>f_{\text{avg}},\\ 1, & f\leq f_{\text{avg}}, \end{array}\right.\\ P_{d}=\left\{\begin{array}{cc} \left(f_{\max}-f\right)\left(f_{\max}-f_{\text{avg}}\right), & f>f_{\text{avg}},\\ 1, & f\leq f_{\text{avg}}. \end{array}\right. \end{array}$$

The experiment uses an arithmetic crossover method to ensure that the resulting offspring are located between the chromosomes of the two parents. In fact, the arithmetic intersection is to perform the following linear combination of random two points *x*_1_ and *x*_2_ in the solution space *D*.

(7) $$\begin{array}{c} \alpha x_{1}+\left(1-\alpha \right)x_{2},\;\alpha \in \left[0,1\right]. \end{array}$$

According to this feature, assuming that *x*_1_ and *x*_2_ represent the parent chromosomes of the crossover calculation, the generated offspring are

(8) $$\begin{array}{c} \left\{\begin{array}{c} x_{1}^{\prime }=\alpha x_{1}+\left(1-\alpha \right)x_{2},\\ x_{2}^{\prime }=\alpha x_{2}+\left(1-\alpha \right)x_{1}. \end{array}\right. \end{array}$$

Chromosomes are encoded by real numbers, and the mutation process is as follows:

(9) $$\begin{array}{c} \left\{\begin{array}{c} x_{1}=x^{\min}-\left|\frac{x^{\min}\times P_{d}\times f}{f_{\max}}\right|,\\ x_{2}=x^{\max}-\left|\frac{x^{\max}\times P_{d}\times f}{f_{\max}}\right|. \end{array}\right. \end{array}$$

The BP neural network uses a three-layer architecture as shown in Figure 1.

The forward computing input is the network output of the output layer, and the input of the JTH node in the hidden layer is

(10) $$\begin{array}{c} {\text{net}}_{j}=\sum_{i}W_{ji}o_{i}+\theta_{j}. \end{array}$$

Among them, *o*_*i*_ is the node input of the input layer *i*, and *W*_*ji*_ is the connection weight between the hidden layer node *j* and the input layer node *i*.

The output analytical expression of the hidden layer node *j* is described as

(11) $$\begin{array}{c} \alpha_{j}=\frac{1}{1+\exp\left({\text{net}}_{j}\right)}. \end{array}$$

The input of the output layer node *k* is

(12) $$\begin{array}{c} y_{k}=\sum_{i}V_{kj}a_{j}. \end{array}$$

Among them, *V* is the connection weight between the output layer node *k* and the hidden layer node *j*.

On this basis, the network deviation function is defined as follows:

(13) $$\begin{array}{c} E=\frac{1}{2}\sum_{k}{\left(t_{k}-y_{k}\right)}^{2}. \end{array}$$

Among them, *t*_*k*_ is the expected output, *y*_*k*_ is the actual output, and *k* is the number of output layer nodes.

The core idea of the BP algorithm is “save the previously calculated results, and then use them for the next calculation, and find the iterative relationship between them, so as to greatly save the computational cost.” The essence of the gradient descent method is to calculate the parameters corresponding to the minimum value of the objective function in the form of iteration. (The objective function is the corresponding error function in deep learning and machine learning.) The core essence of the standard BP algorithm is a kind of optimized algorithm which shows a decreasing grad. And this will lead to oscillations during the learning course and the slowing down in the convergence speed. It is also important to pick up the influencing learning factors. The thesis will take the experiment steps repeatedly till the expected requirement about the accuracy is reached.

The training of the BP network is finished, the collected data from the remote sensor will be dealt with in blocks, and the information integration will be on the way. The model based on the information integration of the genetic neural network is presented in Figure 2.

### 3.3. AHP and Neural Network Landscape Design Effect Evaluation Method

1. Build an ED system for the landscape design. Expert system is an intelligent computer program system, which contains a large number of expert-level knowledge and experience in a certain field. It can apply artificial intelligence technology and computer technology to reason and judge according to the knowledge and experience in the system and simulate the decision-making process of human experts, so as to solve those complex problems that need human experts to deal with.
2. Determine the weight of the landscape design evaluation index using the analytic hierarchy process.
3. Collect landscape design evaluation sample data *v*, use experts to score landscape design evaluation results, and form a landscape design evaluation index sample set.
4. The number of input nodes of the BP neural network is determined by the number of landscape design evaluation indicators, the landscape design evaluation effect is used as the output of the BP neural network, and the number of hidden nodes of the BP neural network is determined according to a certain formula, thereby establishing the BP neural network topology.
5. The related parameters of the BP neural network will be restarted.
6. Employ BP neural network to learn the training samples of landscape design evaluation, and determine the optimal parameters with the accuracy of landscape design evaluation as the training goal.
7. Build a landscape design evaluation model according to the optimal parameters, and use the landscape design evaluation test samples to test the performance of the model.

Based on the above, the specific process of landscape design evaluation of AHP and neural network is shown in Figure 3.

## 4. Analysis of Experimental Results

### 4.1. Analysis of the Model Stability

If the head of the sensor cluster is not changed, with the increasing of the number of the damaged notes, the possibility that the damaged notes turn into the clusters will present a liner rise. Therefore, the probability of it will be regarded as the index of the stability of the model.  Figure 4 shows the ending results.

### 4.2. Analysis of Energy Consumption

As for the information storage and processing, the real number encoding is employed to decrease the consumption of the node information storage. In this experiment, there are 110 nodes in numbers that make up the sensor network lying in the landscape area, and the numbers are distributed in the scope of 110 m× 110 m, which can be presented in Figure 5.

#### 4.2.1. Setting of the Test Environment

In order to test the landscape design evaluation performance of AHP and neural network, specific experiments are used to test their performance. The evaluation environment is shown in Table 1.

#### 4.2.2. Test Object

For the results of 50 landscape design plans, the scores are given by many experts in the same working field who have ranked them in terms of indicators and their experience. The grade will be shown in Figure 6.

From Figure 6, it can be found that the scoring results of different landscape design results are different, showing that the landscape design effects are featured by the certain randomness.

#### 4.2.3. Comparison of the Evaluation Accuracy of the Landscape Index Layer

10 schemes about the design were selected as test samples at random, and the rest ones were used as the training sample ones. Each method was tested for 5 times to reflect the objectiveness of the experimental results. The accuracy of landscape design effect evaluation is demonstrated in Figure 7.

Through the comparison in Figure 7, it can be known that the average accuracy of the method in this paper is 91.52%, the average accuracy of landscape design effect evaluation of AHP is 84.20%, and the average accuracy of landscape design effect evaluation of BP neural network is 86.3%. Compared with the comparison method, the evaluation error of the landscape design effect of the method in this paper is greatly reduced. This is mainly because the method of this paper integrates the advantages of the analytic hierarchy process and neural network and solves the defect of the large error of the current landscape design effect evaluation, which verifies the superiority of the landscape design effect evaluation method in this thesis.

#### 4.2.4. Comparison of Evaluation Efficiency of Landscape Index Layer

The landscape design effect evaluation time of 5 simulation tests for each method is counted, and the results are shown in Figure 8.

It can be seen from Figure 8 that the evaluation time of the landscape design effect of the method in this paper is significantly less than that of the comparison method, which overcomes the shortcomings of the current low efficiency of landscape design effect evaluation and improves the speed.

### 4.3. Urban Landscape Maintenance Management Methods

The completion of garden green space does not mean the completion of the garden landscape “three planting, seven breeding.” We should ensure the sustainability and long-term effectiveness of garden greening and not only do one-time greening projects. If the maintenance work is not done well, the garden landscape built at a great cost cannot be maintained well, and some will soon show grassland degradation, tree death, and overgrown weeds. Therefore, landscape maintenance should implement scientific and standardized scientific maintenance and management. Among many plants, how their later growth conditions are closely related to their conservation and management methods. The general method is basically similar for each region, but for different regions, different types of plants grow in different environments, and the maintenance methods are different. Therefore, in terms of plant maintenance methods, scientific maintenance methods should be selected according to their functions, environment, climate, and soil. For example, climbing plants have different watering levels under different climatic conditions, and the same hedgerows are trimmed in different environments. All are different.  Figure 9 shows the pattern indicators that need to be considered when maintaining and managing urban landscapes.

Plant conservation in the urban environment is not a task that can be accomplished at one time, and long-term and short-term planning must be made according to the urban space, environment, and function. Think carefully about which plants to take and what measures to take. The improvement of plant landscape maintenance can be improved from the following aspects.

One is plant selection and configuration optimization. Plant selection should be suitable for trees in the right place, and on this basis, try to increase plant species, and appropriately introduce exotic plant landscape varieties to enrich the levels and types of green plant landscapes. It is necessary to use vines with climbing ability and good growth from multiple angles. The optimization of plant configuration can increase colorful flowering shrubs, and the lower layer should be combined with drought-tolerant, shallow-rooted succulent herbs. According to the features of Nanjing's urban environment, the plant landscape mostly chooses plants that can reduce noise and have strong adaptability. In terms of plant configuration and maintenance, it is necessary to choose a method that adapts to local conditions, choose native plants as much as possible, pay attention to the matching of plant varieties, and use artistic and aesthetic methods and means to create a comfortable plant landscape.

The second is to establish the concept of overall development from the perspective of long-term planning of plant landscapes and reserve certain planning, three-dimensional and green spaces. The maintenance and management of landscaping must strengthen the scientific management and planning of landscaping projects and strictly follow the norms. Nanjing is a famous ancient cultural capital. Considering the large number of cultural heritages here, the development of Nanjing's ancient culture and the inheritance of new cultures should also be considered, and the cultural heritage spirit of plant landscapes can be added. As an important case of plant landscape design, it is perfectly combined with urban beautification and road greening.

Third, the plant landscape design should fully consider the urban function. Taking the urban road function as an example, different types of road green space and plant landscape need to be combined with specific road functions to configure plants. For example, the three-dimensional greening plant configuration in the traffic island can increase the plants with strong orientation and permeability, which can be used as a guide to guide the plants to choose some plants that do not affect the line of sight. In the plant landscape design of the city square, considering its bearing capacity and the surrounding traffic flow lines, it can be combined with the specific square function, scale, and surrounding environment design, combined with the main body of the square, and the plant configuration can be reasonably arranged to form a transparent and open space.

## 5. Conclusion

Landscaping landscape design is a thinking process and planning strategy for people with relevant professional knowledge of architecture, plants, aesthetics, literature, etc. to consciously transform the natural environment on the basis of traditional garden theory. Through landscape design, the environment has aesthetic appreciation value, daily use function, and can ensure ecological sustainable development. This paper studies the urban landscape design and maintenance management method based on multisource big data fusion. It is necessary to focus on the theoretical research, combine practical conditions, and learn about the latest technologies and application forms of plant landscape maintenance at home and abroad, enrich the variety and resources of plant landscapes, and constantly explore and innovate plant landscape maintenance methods and related maintenance technical issues. In terms of practical basis, it is necessary to strengthen the practical citation of theoretical research, popularize the methods and specialization of plant landscape conservation, and promote the comprehensive and scientific development of the industry [5].

## Figures and Tables

**Figure 1:** BP neural network architecture diagram.

**Figure 2:** Schematic diagram of the information fusion model.

**Figure 3:** The landscape design evaluation process of AHP and neural network.

**Figure 4:** Possibility of damaged nodes leading to cluster heads.

**Figure 5:** Comparison of information fusion energy consumption of three different models.

**Figure 6:** Score values of 50 landscape design effects.

**Figure 7:** Comparison of the accuracy of landscape design effect assessment by different methods.

**Figure 8:** Comparison of landscape design effect assessment time for different methods.

**Figure 9:** Analysis of the urban landscape pattern index system.

**Table 1:** Settings of the test environment.

Type of environment	Parameter	Parameter value
Hardware environment	CPU	AMD 3.0 GHz
	RAM	16 GB
	Hard disk	1000 GB SDD
	Network card	1000 M

Software environment	Operating system	Win 10
	Programming tools	VC 6.0++

## Data Availability

The figures and tables used to support the findings of this study are included in the article.
